RETRACTED

# Evaluation of Chemopreventive Effects of *Acanthus ilicifolius* against Azoxymethane-Induced Aberrant Crypt Foci in the Rat Colon

**DOI:** 10.1371/journal.pone.0096004

**Published:** 2014-05-12

**Authors:** Amel A. Almagrami, Mohammed A. Alshawsh, Riyadh Saif-Ali, Abdrabuh Shwter, Sameer D. Salem, Mahmood A. Abdulla

**Affiliations:** 1 Department of Biomedical Science, Faculty of Medicine, University of Malaya, Kuala Lumpur, Malaysia; 2 Department of Pharmacology, Faculty of Medicine, University of Malaya, Kuala Lumpur, Malaysia; 3 Department of Biochemistry, Faculty of Medicine, Sana'a, Yemen; IIT Research Institute, United States of America

## Abstract

**Background:**

*Acanthus ilicifolius*, a mangrove medicinal plant, is traditionally used to treat a variety of diseases. The aim of this research is to assess the chemoprotective outcomes of *A. ilicifolius* ethanolic extract against azoxymethane (AOM) induced colonic aberrant crypt foci (ACF) in rats.

**Methodology/Principal Findings:**

In our study, rats were arranged in to five groups. Rats in the normal control group were given subcutaneous injections of normal saline once weekly for 2 weeks. The AOM control, reference and treatment groups were given subcutaneous injection of AOM, 15 mg/kg body weight, once weekly for 2 weeks each. The reference group was treated with 35 mg/kg 5-Fluorouracil via intraperitoneal injection once weekly for 8 weeks, and the treatment groups were administered by gavage with 250 and 500 mg/kg *A. ilicifolius* extract daily for 8 weeks. Both normal and AOM control groups received the vehicle; 10% Tween-20 only.

Rats treated with 250 mg/kg and 500 mg/kg of *A. ilicifolius* extracts showed a decrease in the mean number of ACF by 65% and 53%, respectively. Those fed with *A. ilicifolius* showed significantly decreased multiplicity of ACF formations when compared with the results from the AOM control group. The 250 mg/kg *A. ilicifolius* treatment group showed significant decreases in lipid peroxidation MDA levels when compared with the AOM control group. In immunohistochemistry staining, the proliferating nuclear cell antigen (PCNA)-positive cells were significantly higher in the AOM control group than in the *A. ilicifolius*-treated groups. RT-PCR showed that *A. ilicifolius* caused a change in the regulation of apoptosis-related genes expression.

**Conclusion/Significance:**

The results of the current study show that AOM-treated rats receiving oral exposure to *A. ilicifolius* demonstrated a significant decrease in the number of ACF in the colon when compared to AOM-treated rats receiving vehicle only. *A ilicifolius* may be an effective herbal approach for the prevention of AOM-induced ACF in the rat colon.

RETRACTED

## Introduction

Colorectal cancer is the fourth leading cause of cancer deaths worldwide [1], with the incidences of confirmed colorectal cancer rising in many countries [2]. Several epidemiological and experimental studies have indicated that plant products exert a protective influence against this disease, and beneficial effects may be partly attributable to polyphenolic phytochemicals, which have a wide range of pharmacologic properties [3]. One conventional treatment for colorectal cancer is 5-Fluorouracil therapy, which has been in use for the past five decades [4].

Azoxymethane (AOM) and its precursor compound dimethylhydrazine are alkylating agents that cause DNA mutation by binding alkyl or methyl groups to guanine residues, resulting in G to A transition mutations [5]. Aberrant crypt foci (ACF) are putative pre-neoplastic lesions that form in the colons of both animal models and humans [6]. These foci have been used as intermediate biomarkers to rapidly evaluate the chemopreventive potential of several agents, including naturally occurring agents against colon cancer [7]. ACF are hyperproliferative lesions located in the human colon, as well as in carcinogen-treated laboratory models that share others characteristics with colon tumors [8]. In addition, ACF are recognized as colonic carcinogenesis biomarkers as well as alleged precursors of colon cancers [9]. ACF are monoclonal gatherings of phenotypically abnormal crypts, always formed in a dose-dependent way in reaction to carcinogen exposure [10]. Within 6–8 hours of exposure to AOM, crypt progenitor cells undergo apoptosis in response to DNA damage. Progenitor cells that avoid apoptosis then start a proliferative response 48–72 hours later [11]. These foci of aberrant crypts begin monoclonally [12] and arise by a process of incomplete crypt fissioning [13].

*Acanthus ilicifolius* Linn. (Family: Acanthaceae) is a spiny herb of the mangrove variety that is distributed widely throughout Southeast Asia where it is used locally for the treatment of snakebites, rheumatism, paralysis, ulcers, wound healing and asthma [14]. The leaves of *A. ilicifolius* have been reported to exhibit hepatoprotective [15] and tumor-reducing activities [16]. In addition, antioxidant, hepatoprotective, leishmanicidal, tumor reducing and anticancer activities of various extracts of *A. ilicifolius* have been reported [15], [16]. Plant-derived compounds such as flavonoids [17], and terpenes and alkaloids [18] are known to have pharmacological properties including cancer chemopreventive effects and cytotoxicity [19]. The phytochemical literature reveals the presence of 2-benzoxazolinone, lignin glucosides, benzoxazinoideglucosides, flavone glycosides and phenylethanoid glycosides in *A. ilicifolius* [20], [21].

RETRACTED

The aim of this study is to investigate the chemopreventive activity of *A. ilicifolius*, studies were performed to evaluate this agent in the prevention of ACF, a well-established early biomarker of colon carcinogenesis.

## Materials and Methods

### Ethics Statement

This study was approved by the Institutional Animal Care and Use Committee (IACUC), University of Malaya, Malaysia. (Ethic No. PM/07/05/2012/MMA (b) (R). Throughout the experiment, all rats were maintained in accordance with the “Guide for the Care and Use of Laboratory Animals” prepared by the National Academy of Sciences and published by the National Institutes of Health.

### Plant Collection and Extraction

Fresh leaves of *A. ilicifolius* were obtained from Ethno Resources Sdn Bhd, Selangor Malaysia, and all of which were compared with the voucher specimen deposited at the Herbarium of Rimba Ilmu, Institute of Science Biology, University of Malaya, Kuala Lumpur. The leaves were tap-washed, and then oven dried for 7 days, before being subsequently thinly crushed in an electric blender. A fine powder (100 g) of *A. ilicifolius* was drenched in 900 ml of absolute ethanol in a conical flask for 3 days at room temperature. The mixture was filtered with filter paper and evaporated under decreased pressure in a Buchi-type rotary evaporator. The final *A. ilicifolius* dried mass yield was 13.5% (w/w) of dry weight. The dry extract of plant was subsequently dissolved in Tween-20, (10% w/v) and given orally to rats at a dose of 250 or 500 mg/kg body weight.

### Chemicals and Reagents

Azoxymethane was obtained from (Sigma Aldrich; USA) and was used to induce ACF in the rats colons. Chemicals were purchased from Sigma-Aldrich or Fisher unless otherwise noted. AOM was dissolved in normal saline and injected subcutaneously to the animals at a dose of 15 mg/kg body weight. 5-Fluorouracil, purchased from (Calbiochem, USA) was used as a reference drug, this was dissolved in normal saline and injected intraperitoneally to the rats at a dose of 35 mg/kg body weight.

### Determination of Ferric Reducing Antioxidant Power (FRAP) Assay

FRAP assay is designed to quantitatively measure the antioxidant capacity in verity of samples. Therefore, it would be an appropriate technique for determining antioxidant in *A. ilicifolius* extract.

The ferric reducing activity of the plant's extracts were estimated using the method developed by Benzie, with little modification [22]. The reaction mixture involved a 300 mmol/l acetate buffer, 10 mmol/l TPTZ (2,4,6-tripyridyl-s-triazine) in 40 mmol/l of HCl and 20 mmol/l of FeCl_3_.6H_2_O. The working FRAP reagent was freshly prepared by combining 25 ml of acetate buffer, 2.5 ml of TPTZ solution and 2.5 ml of FeCl_3_.6H_2_O. This combination was then incubated at 37°C in water bath for five minutes and then a blank reading was taken spectrophotometrically at 593 nm. After that, 10 µl of standard extract is included to 300 µl of the working FRAP reagent. Absorbance is calculated as happening instantly upon inclusion of the working FRAP reagent after mixing. Thereafter, an absorbance reading was taken four minutes later.

RETRACTED

### Determination of Total Phenolic and Flavonoid Contents

The *A. ilicifolius* extract was evaluated for total phenolic content using Folin-Ciocalteu reagent and was calculated as gallic acid equivalents in mg (GAE)/g of extract according to the Folin-Denis colorimetric method [23]. However, the total flavonoids were determined by using the aluminum chloride colorimetric method, and expressed as quercetin equivalents in mg (QE)/g of extract, as described by Dowd [24]. Both assays were carried out in triplicate.

### Acute Toxicity

Adult male and female Sprague-Dawley (SD) rats (6–8 weeks old and weighing 120–150 g) were obtained from the Animal House, Faculty of Medicine, University of Malaya, Kuala Lumpur. Acute toxicity was performed according to the OECD guideline standard methods [25]. The acute toxicity study was used to determine a safe dose for *A. ilicifolius* extracts. The test extracts should be administered to animals to identify doses causing no adverse effect and doses causing major (life-threatening) toxicity. Thirty-six SD rats (18 males and 18 females) were equally assigned into 3 groups labeled as vehicle (10% Tween-20), low dose (2 g/kg) and high dose (5 g/kg) of *A. ilicifolius* extracts. The animals were fasted overnight (food but not water) prior to dosing. Food was withheld for a further 3 to 4 hours after dosing. The animals were observed at 30 minutes and then 2, 4, 8, 24 and 48 hours after the administration for the onset of clinical or toxicological symptoms. Mortality, if any, was observed over a period of 2 weeks. The animals were sacrificed on the 15^th^ day after fasting overnight. Serum liver and kidney function parameters (Total bilirubin, Direct bilirubin, GOT, GPT, Alk, urea, creatinine) were determined following standard methods, which included histology examinations of the liver and kidneys for any abnormalities.

### Animals and Treatments

Healthy adult SD male rats weighing 120–150 g were obtained from the experimental Animal House, Faculty of Medicine, University of Malaya. The animals were randomly separated into 5 groups of 6 rats each, they were then kept in individual wire-bottomed cages. The animals were given standard rat pellet diet (Altromin; Germany) containing 19% crude protein, 4% crude fat, 6% crude fibre and 7.5% crude ash.

RETRACTED

The experimental design for the present study is shown in Figure 1. The animals were treated as follows:

**Figure 1:** Experimental protocol for AOM-induced colonic aberrant crypt foci formation in male rats. The animals were randomly divided into 5 groups and fed with 10% Tween-20 for the normal control. AOM was given once a week for 2 weeks at a dose of 15 mg/kg of body weight, by subcutaneous injection. 5-Fluorouracil was administered at 35 mg/kg by intraperitoneal injection. *A. ilicifolius* was fed at 250 and 500 mg/kg.

Group 1 (normal control) were given subcutaneous injections of normal saline once weekly for a period of two weeks. Normal control rodents were administered by gavage with 10% Tween-20 for 8 weeks.
Groups 2–5 received subcutaneous injections of AOM, 15 mg/kg body weight, once weekly for 2 weeks.
Group 2, the AOM control group, were administered by gavage with 10% Tween-20 for 8 weeks.
Group 3, the reference group, received intraperitoneal injection of 5-Fluorouracil drug (5-Fu), 35 mg/kg body weight, once weekly for 8 weeks.
Groups 4 and 5 were administered by gavage with 250 and 500 mg/kg A. ilicifolius daily for 8 weeks, respectively.

The body weights of all animals were documented once per week for 10 weeks. All rats were subsequently sacrificed following overnight fasting and under anaesthetic using proper dosages of Ketamine (50–100 mg/kg) and Xylazine (5–10 mg/kg). Blood samples were than gathered; with serum being set apart for examination of biochemical parameters. The colons were washed with cold normal saline and were evaluated for ACF. Colons were slit open lengthwise from the anus to the rectum and then fixed flat with the mucosa on the upper side between layers of filter papers in 10% phosphate-buffered formalin.

### Gross Quantification of ACF in Colon Mucosa

Colons were split open longitudinally and cut into proximal, middle and distal portions of the same length. Topographic examination of the colonic mucosa was performed with Bird's modification [8]: In brief, the colon was fixed in 10% phosphate-buffered formalin for half an hour at 4°C. Next, the colon was stained with 0.2% methylene blue solution for 10 minutes, placed on a microscope slide with the mucosal side upward, and observed under a microscope (10×). The sum of ACF in the entire colon, from the distal to the proximal end, was counted in 2-cm segments. Aberrant crypts were differentiated from the surrounding regular crypts by their enlarged size, increased distance from lamina to basal surfaces of cells, and easily perceptible pericryptal zone. The variable used to evaluate the aberrant crypts foci was the mean number of ACF presented as multiplicity. Aberrant crypt multiplicity was considered to be the number of crypts in every focus and classified as containing up to four or more aberrant crypts/foci. Under light microscopy, a microfeather scalpel blade was used to excise the ACF of interest from the surrounding normal crypts.

RETRACTED

### Histopathological Examination

The colons were dissected into 1 cm×1 cm squares and fixed for 24 hours in 10% buffered formalin solution for histological study. The fixed tissues were processed by automated tissue processing apparatus and embedded in paraffin wax using standard methods. Serial sections of 5 µm thickness were cut parallel to the muscularis mucosa and stained with hematoxylin and eosin. The histology of each ACF was assessed for crypt architecture and nuclear features by comparing them to the normal surrounding crypts.

### Immunochemistry for PCNA

Colon tissues were fixed in 10% buffered formalin and were prepared by an automated tissue processing machine. Colon samples were also embedded with paraffin. Sections (3–5 µm) were mounted on to poly-L-lysine covered slips and positioned in an oven (Venticell, MMM, Einrichtungen. Germany) at 60°C for two hours. The sections were deparaffinised, hydrated, and exposed to antigen retrieval by immersion in 10 mM citrate buffer (pH 6.0) that was boiled in a microwave at 92–95°C for 20 minutes. Immunohistochemistry staining steps were performed following the manufacturer's instructions (Dako Cytomation, USA). In brief, endogenous peroxidase was blocked using 0.03% hydrogen peroxide sodium azide for 5 minutes. Tissue sections were washed gently with wash buffer and then incubated with Proliferating Cell Nuclear Antigen (PCNA) (1∶200) biotinylated primary antibodies for 15 minutes. Sections were gently washed with wash buffer and kept in the buffer bath in a humid chamber. A sufficient amount of streptavidin- HRP was then added and incubated for 15 minutes followed by washing. Diaminobenzidine substrate chromagen was added to the sections and incubated for over 7 minutes followed by washing and counterstaining with hematoxylin for 5 seconds. The sections were then dipped in weak ammonia (0.037 M/L) 10 times, washed and cover slipped.

All sections were observed under light microscopy and were evaluated by an observer who was blinded to the experimental protocol. Positive antigens stained brown under light microscopy. Five independent sections of the colon from each rat were stained, and 1,500 cells were measured from every area. The PCNA marking (PI) was calculated as the [(number of positive cells)/(total number of epithelial cells)]×100 for each area. These PI values for all the different colon sections of the rats belonging to the same group were then averaged.

RETRACTED

### Estimation of Lipid Peroxidation Level in Colon Tissue

Colon samples were rinsed instantly with cold saline to remove as much blood as possible. Colon homogenates (10% w/v) were arranged in cold 50 mM PBS (pH 7.4) using homogenizer in ice. Cell particles were eliminated by centrifugation in a refrigerated centrifuge at 4500 rpm for 15 minutes at 4°C. The supernatant was used for the estimation of the lipid peroxidation level using a commercially available malondialdehyde (MDA) kit (Cayman Chemical Company, USA): Briefly, MDA levels were measured in the colon tissue homogenate of all experimental groups as a measure for lipid peroxidation, using thiobarbituric acid. Ready-to-use SDS solution was added (100 µl) to the samples/standard (100 µl). Next, 4 ml of color reagent was added to the mixture. Samples and standard solution tubes were immersed in boiling water for 1 hour. The reaction was stopped by incubation in an ice bath for 10 minutes. All tubes were then centrifuged at 1600×g for 10 min at 4°C. A set of duplicate samples or standards were loaded into a 96-well plate, and the absorbances were read at 532 nm with a plate reader.

### Real-Time Quantitative Polymerase Chain Reaction Analysis

Colon samples were immediately placed in RNA *later* Solution (Ambion, USA) incubated over night at 4°C and stored at −80°C. Total RNA was isolated according to the manufacturer's instructions using RNeasy plus Mini Kits (cataloge No74134, Qiagen, Germantown, Maryland, USA) on the homogenized tissue of the treated and untreated rats. RNA concentrations were measured by a Nano Drop ND-2000 spectrophotometer (Thermo Fisher, USA). RNA quality and integrity were concluded through the A260/A280 ratio and agarose gel electrophoresis respectively. One microgram of total RNA was transcribed to cDNA using a high capacity RNA-to-cDNA reagent from (Applied Biosystems, USA). cDNA synthesis was used as suggested by the manufacturer. RT-PCR was carried out by ABI TaqMan gene expression assays for Bcl-2 (assay ID: Rn99999125), Bax (assay ID: Rn02532082), and p53 (assay ID: Rn00755717) according to protocol guidelines. All samples were run in triplicate in total reaction volume 20 µl: 10 µl master mix, 1 µl TaqMan gene expression assay 2 µl cDNA, and 7 µl Nuclease-free water.

Quantitative RT-PCR was performed using TaqMan fast advanced master mix (Applied Biosystems, USA) and the step one plus Real Time PCR system (Applied Biosystems, USA) in triplicate wells. The cycle parameters were as follows: activation at 95°C for 20 s, 40 cycles of denaturation at 95°C for 1 s, and then annealing and extension at 60°C for 20 s. The data was analysed using a comparative threshold cycle (Ct) technique. Gene expressions were calculated using Gene Ex software (MultiD Analyses AB, Sweden). The corresponding mRNA level from colonic mucosa of the normal group (calibrator) was used as an external reference. The levels of Hprt1 (assay ID: Rn01527840) and Tbp (assay ID: Rn01455646) mRNA were used as an internal reference to standardize the data. The fold changes of each mRNA (mRNA relative expression) were expressed relatively to the mean value of the related mRNA located in the mucosa of the normal control rats and was calculated using the ^2-ΔΔ^Ct method.

RETRACTED

### Statistical Analysis

The statistical analysis was performed using the one-way analysis of variance (ANOVA) technique followed by a post hoc test with Bonferroni's multiple comparison equation. All values were calculated as the mean ± SEM. A value of *p*<0.05 as compared to the respective AOM control group was considered significant.

Real-time PCR data was analysed by using GenEx program version 5.4 (GenEx program, www.multid.se). Fold changes were calculated and T-test was used to evaluate the difference between groups for all genes. *P*<0.05 was considered as significant.

## Results

### Acute Toxicity Study

In the acute toxicity study, animals were treated with the *A. ilicifolius* extract at doses of 2 g/kg and 5 g/kg and whilst being kept under observation for 14 days. All the animals remained alive, and none manifested any significant visible toxicity at these doses. There were no abnormal signs, behavioral changes or body weight changes. There was no mortality observed at the above-mentioned doses by the end of the 14 days of observation. Serum liver and kidney function parameters revealed no significant differences between treated and untreated groups. Moreover, liver and kidney histology examination confirm that there were no abnormalities present. As a result, it was concluded that the extract induced no mortality and no evidence of either hepatic or renal damage following a single dose of up to 5 g/kg.

### Ferric-Reducing Antioxidant Power (FRAP) Assay Results

Figure 2 reveals that 1 mg/ml of *A. ilicifolius* has a strong reducing power as it significantly (*p*<0.05) with greater FRAP value 1670±0.277 µmol Fe II/g in comparison to BHT and vitamin C (1 mg/ml) were the FRAP value 521.4±0.82 and 1181.9±0.274 µmol Fe II/g respectively. Furthermore, the FRAP value for the quercetin and gallic acid (1 mg/ml) were revealed to be 2267.1±0.55 and 2640±0.277 µmol Fe II/g respectively.

RETRACTED

**Figure 2:** Ferric reducing activity of *A. ilicifolius* extract. All values are expressed as mean ± SEM. Mean with different letters indicate significantly different values *P*<0.05. BHT; Butylatedhydroxyl toluene.

### Total Phenolic and Flavonoids Contents

The total phenolic content of the ethanolic extract of *A. ilicifolius* was 281.90±0.27 mg (gallic acid equivalents) per g of extracts with the standard curve equation: *y* = 0.0007*x*+0.0015, *R* ^2^ = 0.989. The total flavonoids were 46.79±0.005 mg (quercetin equivalents) per g of extracts (the standard curve equation: *y* = 0.0054*x*+0.005, *R* ^2^ = 0.999), and the ratio of flavonoids/phenolic was 0.2. Thus, phenolic compounds were the predominant antioxidant components in *A. ilicifolius* extracts, leading to more potent scavenging of radicals.

### Efficacy of *A. ilicifolius* on ACF Formations

ACF were mostly observed in the middle colon. ACF in the colon were counted, and the total numbers of ACF and of crypts per focus were averaged. ACF were observed in the colon, as well as in multi-crypt clusters (which contained a multiplicity of crypts/foci) of aberrant crypts (Table 1). Rats treated with AOM and fed with the low and high doses of *A. ilicifolius* extract showed a significant reduction in the total ACF/colon compared with AOM control rats, to the extent of 65% and 53% inhibition respectively (*P*<0.0001). The multiplicity of aberrant crypts/foci were also significantly reduced in rats fed with *A. ilicifolius* when contrasted with AOM-induced rats (*P*<0.0001).

**Table 1:** Inhibitory effects of *A. ilicifolius* on AOM-induced multiplicity of aberrant crypt foci in rat colon.

Groups	1 crypt	2 crypts	3 crypts	4 crypts	5 & more crypts	Total ACF	Conc.of
							inhibition
AOM control	19.50±3.62	29.79±4.89	23.04±2.70	24.67±2.22	34.33±4.94	131.33±15.09	0
							
5-Fluorouracil	10.1667±1.04	9.50±2.04*	7.91±.69**	6.25±.81**	7±.64**	40.83±3.06**	69%
							
LD 250 mg/kg	18.36±3.14	10.05±1.63*	4.30±.0.16**	4.47±.0.57**	8.13±0.89**	45.33±4.43**	65%
							
HD500 mg/kg	17.08 ±2.37	13.08±2.55	11.91±.0.95**	8.75±.0.86**	9.08±1.55**	62±3.72**	53%
							

Values are expressed as the mean ± SEM.;

^*^ *P*<0.001 *versus* AOM control group and;

^**^ *P*<0.0001 *versus* AOM control group.

### Macroscopic Findings

As presented in Figure 3, the AOM-control rats developed grossly identifiable ACF in the colon. No aberrant crypts were identified with methylene blue in the intact colons of normal control rats. The multiplicity of ACF, are considered to be precursor lesions to colon cancer, was significantly higher in AOM group compared to *A. ilicifolius*-treated groups.

RETRACTED

**Figure 3:** Effects of *A. ilicifolius* on AOM-induced ACF in rat colon. Topographic views of ACF in methylene blue staining of rat colonic tissue showing: (A) Normal crypts from rats treated with 10% Tween 20, normal control. (B) AOM control group, with significant increases in the ACF numbers. (C) Reference group (5-Fluorouracil) + AOM. (D) 250 mg/kg *A. ilicifolius* + AOM. (E) 500 mg/kg *A. ilicifolius* + AOM. (10×).

### Histopathology Examination

Histological sections of ACF were cut parallel to the muscular layer. Tissue sections of all grossly visible AFC on colon mucosa were stained with hematoxylin and eosin stains in order to be evaluated. The normal control group showed circular shapes and basal location of the nuclei. The AOM control group contained comparatively more ACF, exhibiting marked nuclear atypia, significantly decreased goblet cells, mucin depletion and narrow lumen. ACF are longer and larger than normal crypts, and the cytoplasm is intensely stained. The epithelial cells in ACF have distinctive elongated and slightly stratified nuclei, loss of cell polarity and an increase in mitosis compared to the surrounding regular crypts (Figure 4). *A. ilicifolius* fed groups showed an increase in apoptosis, reduced mitosis and cellular proliferation, a reduced induction of ACF in the rats colons, with only mild morphological changes associated with ACF when compared with the AOM-treated group (cancer control).

**Figure 4:** Effects of *A. ilicifolius* on histological sections of AOM-induced ACF. All sections were cut parallel to the muscular layer. (A) Normal colon mucosa showing circular shape of the crypts and nuclei lining the crypt, basal nuclear polarity and absence of stratification. (B) AOM treated group showed elongated ACF with narrow lumen, marked nuclear atypia (elongated and stratified nucleus), loss of basal nuclear polarity and increases proliferation with decreases in goblet cells (C) Reference group, 5-Fluorouracil + AOM showed slightly elongated ACF and nuclei, slight decreased in goblet cells and no nuclear stratification. (D) 250 mg/kg A. ilicifolius + AOM showed elongated ACF and nuclei, slight decreases in goblet cells and nuclei showed slightly nuclear stratification (E) 500 mg/kg A. ilicifolius + AOM showed ACF with slightly rounded shape and without stratified nuclei, slightly decreased in number of goblet cells and proliferation of nuclei (H & E stain 100×).

### Effects of *A. ilicifolius* on PCNA Staining of Colons and Cell Counting in AOM-Induced ACF in Rats

PCNA was evaluated as a marker for cell proliferation in the colon specimens. Sections of colon samples from the control group and *A. ilicifolius*-treated groups are shown (Figure 5). The PCNA staining (brown red) of cell nuclei of colon mucosa was much stronger in AOM control rats than in *A. ilicifolius*-treated rats. PCNA-negative cells (blue) were stained with hematoxylin. The PCNA labelling index is also shown in (Figure 6). The colon sections from the AOM control group exhibited a significantly higher number of positive cells than those sections from the *A. ilicifolius*-treated group. The percentage of PCNA-positive cells of colon mucosa in normal control group were 3.4±0.1%, whereas the percentage of PCNA-positive cells in AOM control group were 48.5±2.5%, 5-fluorouracil 11.67±1.03%, low and high-doses of *A. ilicifolius*- treated groups were 28.2±2.75% and 33.6±2.82%, respectively.

RETRACTED

**Figure 5:** Effects of *A. ilicifolius* on PCNA Staining. All sections were cut parallel to the muscular layer. The immunohistochemical staining method was used to detect PCNA-labelling indices (PI) in specimens with AOM-induced ACF in colon tissue including those fed with *A. ilicifolius*. PCNA-negative cells were (stained blue) and PCNA positive cells were (stained brown). PCNA was evaluated as a marker for cell proliferation in the colon specimens. Sections of colon samples from the control group and *A. ilicifolius*-treated groups. The PCNA labelling index (PI) was calculated as the [(number of positive cells)/(total number of epithelial cells)]×100 for each field. (A) Normal control group showed significantly lower PCNA indices compared to AOM control group (arrow). (B) AOM-control group showed significantly higher PCNA indices than those in groups C, D, and E (arrow). (C) 5-Fluorouracil (standard drug)-fed group + AOM showed significantly lower PCNA indices than AOM-control group. (D) Rats fed with 250 mg/kg *A. ilicifolius* + AOM, showed significantly lower PCNA indices than the AOM control group (arrow). (E) Rats fed with 500 mg/kg *A. ilicifolius* + AOM showed significantly lower PCNA indices than AOM-control group (Immunohistochemical (PCNA) staining X100).

**Figure 6:** Effects of *A. ilicifolius* on PCNA counting. All values are expressed as the mean ± SEM. *  =  significantly different means compared to the AOM group, mean with #  =  significantly different means compared to the normal group, *p*<0.01.

### Effects of *A. ilicifolius* on Lipid Peroxidation Level in AOM-Induced ACF in Rats

Treatments of both doses of *A. ilicifolius* reduced the lipid peroxidation (MDA) level compared to the higher level generated in the AOM control group however the lower dose (250 mg/kg) was the one which most significantly reduced amounts of MDA. The lipid peroxidation (MDA level) was significantly higher in the AOM group compared to the normal control group and treatment groups. Feeding AOM-treated rats with 250 mg/kg of *A. ilicifolius* significantly reduced the lipid peroxidation level, to a near normal state. Thus, treatment with either *A. ilicifolius* extract or 5-Fluorouracil reduced the toxicity of AOM, as shown in (Figure 7).

RETRACTED

**Figure 7:** Effect of *A. ilicifolius* extract on lipid peroxidation level. All values are expressed as the mean ± SEM. Significant differences have values of *P*<0.05.

### Effect of *A. ilicifolius* on Apoptosis Gene Expression

Treatments with *A. ilicifolius* significantly upregulated the expression level of proapoptotic Bax gene and p53 protein in the mucosa of the AOM-injected rats. Bcl-2 gene expression levels showed no significant change due to exposure to *A. ilicifolius* treatment. The deregulation of crypt cellular proliferation in the colon of the AOM-injected rats was associated with (Bcl-2/Bax >1), while the upregulation of Bax in *A. ilicifolius* treatment groups caused a change in the Bcl-2/Bax ratio value which was reserved to (Bcl-2/Bax <1) (Figure 8).

**Figure 8:** Changes in the mRNA Expression Levels of Bax, Bcl-2 and p53. Data are presented as the mean ± SEM, *P*<0.05.

## Discussion

Practitioners of traditional herbal medicine have described the supposed therapeutic effects of many indigenous plants for various diseases [26]. Natural products are a source of both synthetic and traditional herbal medicine which remain the primary health care system in some parts of the world [27]. Plant resources, namely vegetables, fruits and spices, have attracted extensive study because of their chemoprotective properties. Many are known to possess anti-inflammatory, antioxidant, antitumor and cancer chemoprevention activities [28]. The AOM-induced colon carcinogenesis model represents a valuable approach for the development of strategies for chemoprevention. This model recapitulates many of the clinical, pathological and molecular features occurring in human colorectal cancer (in around 80% of cases), including crypt cell hyper-proliferation and ACF formation, which are considered premalignant precursors [29]. Preneoplastic lesions such as ACF, which are detected 30–45 days after AOM administration, have been extensively used as an endpoint in short-term chemopreventive studies [7]. In fact, ACF are considered to be the ‘gold standard’ in terms of colon carcinogenesis biomarkers [9].

The antioxidant effects of various extracts of *A. ilicifolius* have been reported previously [15], [16]. Furthermore, a number of studies have shown a relationship between oxidative stress and carcinogenesis. Free radicals, which are able to either directly damage DNA or enhance the genetic instability of affected cells, can thus be involved in the first stage of neoplastic transformation, called *initiation* [30].

RETRACTED

Phenolic antioxidants are essential for the human body to remove and naturalize the free radicals that are otherwise present. Many polyphenols, such as flavonoids, have been identified as being highly effective antioxidants; they also perform a significant role in the treatment of many diseases. In experimental animal models, azoxymethane (AOM) increases the oxidative stress of colon cells, which then develops into colon cancer in rats [31], [32].

Our study showed that treatment of animals with 250 mg/kg *A. ilicifolius* significantly reduced the lipid peroxidation (MDA) level compared to the high level generated in the AOM control group, which might be due to the high total phenolic and flavonoid contents in the *A. ilicifolius* plant. In contrast, AOM significantly enhanced the MDA level compared to the normal control group. Treatment of animals with *A. ilicifolius* extracts and 5-Fluorouracil significantly reduced the levels of MDA and lipid peroxidation. The results of the current study are in agreement with the findings of Shahidi and Chandrasekara that suggest chemopreventive effects could be linked to their capability to decrease free radical development and to scavenge free radicals [33]. Similarly, previous studies have established that enhancing the activities of antioxidant enzymes (superoxide dismutase and catalase) reduces AOM-induced colon cancer in animals, suggesting that the reduction of oxidative stress likely plays a role in the mechanism of its chemopreventive effects [34].

In the present study, we show that feeding rats with *A. ilicifolius* at 250 mg/kg or 500 mg/kg reduced the numbers of foci containing 3 or more aberrant crypts/foci. This plant considerably decreased total colonic AOM-induced ACF formation and multicrypt aberrant crypt growth. *A. ilicifolius* was observed to be effective in inhibiting ACF, and it is possible that this plant may provide some antioxidant activities that contribute to the prevention of carcinogenesis, as previously reported [15], [16]. A large number of antitumor agents obtained from plants exhibited their effects through apoptosis induction in cancer cells [35]. A Few of the previous studies involving naturally occurring agents, such as curcumin [36], caffeic acid [37], and diosgenin [38], considerably suppressed AOM-induced colon ACF as well as colon adenocarcinoma in male rats. Likewise, administration of *A. ilicifolius c*an significantly decrease the occurrence of ACF in rat colon.

RETRACTED

Consistent with our study, Tanaka found that an orange juice phytochemical, hesperidin, might inhibit the ‘initiation phase’ of colon carcinogenesis. Moreover, Tanaka noted that the inhibition of carcinogenesis by hesperidin was partly due to decreased cell proliferation in the colonic mucosa [39]. In contrast to the results of the present study, pectin increased chemically induced colon cancer [40].

Colon carcinogenesis is a multistage process, with quick cell proliferation and ablation of apoptosis as initial incidences for its progression [41]. Cell proliferation and apoptosis biomarkers are generally used to examine the efficacy of potential chemopreventive agents [42]. Several studies involving human and animal models showed that one of the earliest indications of preneoplasia is abnormal epithelial cell proliferation, maturation and differentiation [43]. Increased cell proliferation has long been shown to play a crucial role in the initiation phase, as well as the promotion/progression stages of carcinogenesis. In this regard, PCNA is suggested as being a factor in DNA replication by developing a moving foundation that could mediate the interaction of numerous proteins with DNA, herefore, PCNA is considered an efficient biomarker for cell proliferation [44]. In the present study, *A. ilicifolius* at either treatment level significantly reduced the increase in the percentages of PCNA-positive cells seen in rats treated with AOM.

In living animals, a regular enhance in ROS can enhance mobile development and differences, however, excessive amounts of ROS can cause oxidative damage to tissues, and may also represent danger in the form of cancer cells [45]. Mitochondria are a source of ROS and execute a main role in the control of apoptotic signalling ROS, as a second messenger in several signalling pathways, plays a significant role in apoptosis by managing the activities of certain enzymes involved in the cellular deaths pathway. [46]. Some anticancer drugs have been exposed to generate apoptosis in tumor cells, in aspect by resulting in the development of ROS [47].

Bcl-2 near family members proteins are made up of two types, pro-apoptotic proteins such as Bax and antiapoptotic proteins such as Bcl-2 [48]. Previous researches have verified that Bcl-2 and Bax recognize in the mitochondrial outer-membrane and the Bcl-2/Bax ratio can be determined as being a key factor in recognizing of the apoptotic process, due to regulating the release of mitochondrial cytochrome c to cytosol [49]. The carcinogenic process needs variations in the balance between cellular recovery and cellular deaths that control frequent cellular homeostasis in the colonic mucosa [50].

RETRACTED

In this study, the deregulation of crypt cellular proliferation in the colon of the AOM-injected rats was associated with the Bcl-2/Bax value (ratio >1). *A. ilicifolius* treatment induced an important upregulation of proapoptotic Bax gene and p53 protein expression leading to a reversal of the Bcl-2/Bax amount (Bcl-2/Bax <1). This type of switch has been formerly exposed in the mucosa of AOM-injected rats after long-term treatment with aspirin drugs, another effective chemopreventive agent for colon cancer prevention [51]. These results agree with those obtained by Bousserouel *et al* [52]. The tumour suppressor protein p53 is known to play an important role in apoptosis and cell cycle arrest [53]. A previously conducted study proved that p53 up-regulated bcl-2 gene expression [52]. Similarly, Bax has previously been determined to be a p53 early-response gene [54], an a exclusive p53 regulated gene which activated apoptosis [55], whilst Bcl-2 is a known apoptosis antagonist [56], [57]. Therefore, these results indicate that treatment with *A. ilicifolius* induced cellular deaths in mitochondrial apoptosis pathways. In addition, the changes in expression of apoptosis-related genes such as the Bcl-2/Bax ratio (antiapoptotic in comparison to proapoptotic gene and protein levels) can be used as indicators and symptoms of chemopreventive efficiency. In conclusion, this study demonstrated that *A. ilicifolius* ethanol extract has high phenolic and flavonoid contents. The extract is toxicologically safe *in vivo* by oral administration, and it has chemopreventive effects against AOM-induced colon cancer that were proven macroscopically, histopathology and through immunohistochemical staining. Accordingly, this plant extract might be an effective herbal remedy against chemically induced colorectal cancer.

## Supporting Information

Figure S1 Total Phenolic Content (TPC) standard curve of the ethanolic extract of *A. ilicifolius*.
(DOCX)

Figure S2 The total flavonoids standard curve of the ethanolic extract of *A. ilicifolius*.
(DOCX)
